# Correlation of Choroidal Thickness and Volume Measurements with Axial Length and Age Using Swept Source Optical Coherence Tomography and Optical Low-Coherence Reflectometry

**DOI:** 10.1155/2014/639160

**Published:** 2014-06-12

**Authors:** Janusz Michalewski, Zofia Michalewska, Zofia Nawrocka, Maciej Bednarski, Jerzy Nawrocki

**Affiliations:** Ophthalmic Clinic Jasne Blonia, ul. Rojna 90, 91-162 Lodz, Poland

## Abstract

*Purpose*. To report choroidal thickness and volume in healthy eyes using swept source optical coherence tomography (SS-OCT). *Methods*. A prospective observational study of 122 patients examined with swept source OCT (DRI-OCT, Topcon, Japan). In each eye, we performed 256 horizontal scans, 12 mm in length and centered on the fovea. We calculated choroidal thickness manually with a built-in caliper and automatically using DRI-OCT mapping software. Choroidal volume was also automatically calculated. We measured axial length with optical low-coherence reflectometry (Lenstar LS 900, Haag-Streit, Switzerland). *Results*. The choroid has focally increased thickness under the fovea. Choroid was thinnest in the outer nasal quadrant. In stepwise regression analysis, age was estimated as the most significant factor correlating with decreased choroidal thickness (*F* = 23.146, *P* < 0.001) followed by axial length (*F* = 4.902, *P* = 0.03). Refractive error was not statistically significant (*F* = 1.16, *P* = 0.28). *Conclusions*. SS-OCT is the first commercially available system that can automatically create choroidal thickness and volume maps. Choroidal thickness is increased at the fovea and is thinnest nasally. Age and axial length are critical for the estimation of choroidal thickness and volume. Choroidal measurements derived from SS-OCT images have potential value for objectively documenting disease-related choroidal thickness abnormalities and monitoring progressive changes over time.

## 1. Introduction

The choroid is a vascular layer that supplies the retina with oxygen and nutrition. Until recently, the only diagnostic tool for visualization of choroid was indocyanine angiography. This is an invasive intervention and can only present blood flow and not histological sections. Optical coherence tomography (OCT) devices were primarily designed to visualize the retina and did not reveal structures lying beneath the retinal pigment epithelium due to light scattering on choroidal vasculature. The function of the choroid is associated with many diseases affecting the retina. Thus, imaging and quantitative assessment of choroidal tissue may be of value for the diagnosis of many retinal and choroidal diseases. Spaide et al., using spectral domain OCT (SD-OCT), (Spectralis OCT Heidelberg Engineering, Heidelberg, Germany), was the first to present that SD-OCT may enable the creation of an inverted image when the device is moved closer to the eye. Since SD-OCT has the highest sensitivity near to zero-delay and sensitivity decreases for larger delays, by inverting the OCT image, the choroid is closer to the zero-delay line, providing enhanced sensitivity and increased imaging depth. The device was called EDI-OCT (enhanced depth OCT) [1]. Other authors have confirmed this observation using other commercially available SD-OCT devices [2]. The inverted image in SD-OCT enables measurement of the choroid at several points. However, the system cannot create 3-dimensional choroid maps as the choroidoscleral boundary may not be detected in all cases due to scattering and low penetration through the RPE, which is influenced by the wavelength used. Some authors attempted to measure choroidal thickness and volume after manual choroidal segmentation [3]. This is perhaps too time-consuming and too complicated for everyday ophthalmic practice. The ability to create choroidal maps, with repeatability similar to the way current SD-OCT devices enable the creation of retina maps, could enable us to precisely determine the mean choroidal thickness in healthy subjects and possibly add information to the pathogenesis and course of various retinal diseases. To produce repeatable choroidal maps, we need exact delineation of the outer choroidal layer, which may be obtained by using a longer light wavelength [4].

The commercially available swept source OCT (SS-OCT; DRI-OCT, Topcon, Japan) uses a longer wavelength than SD-OCT (1050 nm versus 840 nm). Longer wavelengths overcome much of the scattering of light on choroidal vasculature, thus it enables a more exact visualization of the choroid. The purpose of the current study was to determine choroidal thickness and volume in healthy subjects with a commercially available SS-OCT device, furthermore, to correlate the results with age, refractive error, and axial length measured with optical low-coherence reflectometry.

## 2. Material and Methods

We included into this prospective study 122 eyes of 122 healthy volunteers with no visual symptoms or history of ocular disease. The Institutional Ethics Committee Board approved the design of the study. The study is also in adherence with the Declaration of Helsinki. All patients had a comprehensive ophthalmic examination. We carried out OCT imaging using the first commercially available SS-OCT device (DRI-OCT, Topcon, Japan) with a wavelength of 1024 nm and used optical low-coherence reflectometry to measure axial length by optical biometry (Lenstar LS 900, Haag-Streit, Switzerland). Axial length measurement is reportedly very precise with this device, as it is based on a similar mechanism to time domain OCT [5]. We measured spherical equivalent refractive error with an Auto Refractometer (NIDEK Co., Ltd., Japan).

Only patients with no abnormalities both in ophthalmic examination and in SS-OCT were included in the current analysis. Patients with a high refractive error were also included. To exclude diurnal variations all examinations were performed at the same time (3–6 pm). It was estimated in earlier studies that axial length is stable during this time period, lower than that at noon and higher than that in the evening [6].

In all cases, two experienced examiners performed two scanning protocols. First, for manual estimation of choroidal thickness we took a single line scan with a resolution of 3 *μ*m, built from 1024 A-scans with a length of 12 mm. Second, we carried out a 3-dimensional scanning protocol with 3 *μ*m axial resolution and a speed of 100,000 A-scans per second. In this protocol, 256 B-scans were taken on an area of 12 × 9 *μ*m.

We took manual choroidal thickness measurements between the line representing retinal pigment epithelium, the outer most hyperreflective retinal layer, and the line representing lamina suprachoroidea, the outer hyperreflective line of the choroid. The caliper used for manual segmentation was included in the software. Black on white images were analyzed to exactly spot the outer choroidoscleral boundary (Figure 1(a)).

We utilized the built-in choroidal segmentation tool to automatically define the outer border of the choroid and measured choroidal thickness between the lines indicating retinal pigment epithelium and the choroidoscleral boundary (lamina suprachoroidea) [7]. Choroidal thickness and volume were automatically calculated using the built-in software (Figure 1). We calculated numeric averages of the measurements for each of the 9 map sectors defined by the early treatment diabetic retinopathy study (ETDRS) [8]. The inner and outer rings with diameters of 3 mm and 6 mm, respectively, were segmented into 4 quadrants. Mean choroidal thickness at the fovea was defined as the average thickness in the central 1000 *μ*m diameter of the early treatment diabetic retinopathy study layout (Figure 1(b)).

Using linear regression analysis and stepwise multiple regression analysis, we investigated the relationship between foveal choroidal thickness and age, sex, spherical equivalent of the refractive error, and axial length. ANOVA on ranks test was performed to compare choroidal thickness and volume in different quadrants. We performed statistical analysis with commercially available software (SigmaStat 3.5 for Windows).

## 3. Results

The current study included 122 eyes of 122 healthy volunteers. Their mean age was 43 years (15–79 years, SD: 17 years); 52 subjects were male and 70 were female. Spherical equivalents varied from −22 diopter to +6 diopter. 27 eyes were emmetropic, 85 eyes were myopic (44 had high myopia: considered as spherical equivalent >6 D), and 10 eyes were hyperopic. The mean axial length measured with optical low-coherence reflectometry was 25.07 mm (21.33 mm–31.04 mm; SD: 2.19 mm).

### 3.1. Choroidal Thickness

Table 1 shows the mean choroidal thicknesses by sector.

Fovea thickness measured manually was significantly thicker than when measured automatically (*P* = 0.04), which may be explained by the fact that the manual measurement is a focal measurement and that the automatic measurement measures the mean thickness in a circle with a diameter of 1000 *μ*m. In eyes with high myopia the automatic and manual measurements did not differ (*P* = 0.42), which may be explained by the lack of focal central increased choroidal thickness in high myopia.

Focal measurements of foveal choroidal thickness were significantly thicker than when automatically measured in all quadrants (*P* < 0.001). Automatically measured foveal choroidal thickness did not significantly differ from any quadrant in the inner ring (inferior quadrant: *P* = 0.4, superior quadrant *P* = 0.8, nasal quadrant: *P* = 0.08, and temporal quadrant *P* = 0.59) but it was significantly thicker than the nasal quadrant in the outer ring (inferior quadrant *P* = 0.2, superior quadrant *P* = 0.3, nasal quadrant: *P* < 0.001, and temporal quadrant *P* = 0.57). Also in the inner ring the choroid was not statistically different on any side of the fovea (nasal versus temporal: *P* = 0.727; inferior versus superior: *P* = 0.293). In the outer ring, the choroid nasal to the fovea was thinner than inferior to the fovea (*P* = 0.034), superior to the fovea (*P* < 0.001), and on the temporal side (*P* < 0.001).

### 3.2. Choroidal Volume

Choroidal volumes in the outer temporal, superior, and inferior quadrant are bigger than in the outer nasal quadrant (*P* < 0.001).  Table 2 shows the mean choroidal volume by sector.

Central choroidal volume was significantly smaller than in all quadrants of the inner and outer rings (*P* < 0.001). However, choroidal volume in different ETDRS subfields is measured from different geometrical figures. Choroidal volume in the fovea is the volume of a cylinder with an upper and lower diameter of 1000 *μ*m and the height of the cylinder is the foveal choroidal thickness (*V* = *πr* ^2^ *h*; *V*—cylinder volume, *r*—radius, and *h*—height). Choroidal volumes in the inner and outer quadrants are volumes of irregular geometrical figures with base diameters bigger than the foveal, which explains why the choroidal volume values in all subfields are bigger than in the center and that they should not be compared directly. What we can separately compare are the values in the inner circle and the values in the outer circle. In the inner circle no statistical difference was observed between particular subfields (Kruskal-Wallis one-way analysis of variance on ranks; *P* = 0.2, *H* = 4.071). In the outer circle the nasal subfield had significantly lower volume than all other subfields (Tukey's test, *P* < 0.05).

### 3.3. Adequacy of the Automated Segmentation

In all cases the examiner was able to estimate the outer choroidal boundary. However in 16% of cases a discrepancy existed between the examiners estimation and the automated measurement. In those cases the automatically drawn lines were manually corrected by the examiners.

### 3.4. Relation to Sex, Age, Refractive Error, and Axial Length

Sex was not found to significantly influence choroidal thickness in the whole group (*P* = 0.47).

Age was found to be negatively correlated with central choroidal thickness (both when automatically measured and manually measured; *P* < 0.001) and with central choroidal volume (*P* < 0.001). Regression analysis revealed that choroidal thickness decreases 1.289 *μ*m each year *R* ^2^ = 0.08 (Figure 2).

Choroidal thickness and volume are also negatively statistically significant dependent on the refractive error (*P* < 0.001). Regression analysis showed that choroidal thickness decreases 12.7 *μ*m with each diopter (*R* ^2^ = 0.25).

Axial length measured with low-coherence reflectometry was also found to be negatively correlated with choroidal thickness and volume (*P* < 0.001). Regression analysis shows that choroidal thickness decreases 28 *μ*m with each mm of axial length (*R* ^2^ = 0.3) (Figure 3).

We also performed stepwise multiple regression analysis to calculate which of the factors, age, axial length and refractive error, are associated the most with choroidal thickness. Age was estimated as the most significant factor (*F* = 23.146, *P* < 0.001) followed by axial length (*F* = 4.902, *P* = 0.03). Refractive error showed no significant association with choroidal thickness in multiple regression analysis (*F* = 1.16, *P* = 0.28).

Stepwise regression analysis also revealed that foveal choroidal volume can be predicted from a linear combination of two independent variables among the above mentioned factors: age (*F* = 22.711, *P* < 0.001) and axial length (*F* = 39.366, *P* < 0.001). Refractive error was not estimated as an independent factor in the stepwise regression analysis (*F* = 2.952, *P* = 0.08).

## 4. Discussion

The Topcon DRI-OCT machine we used was the first commercially available device of its kind. It enables automatic creation of choroidal volume and thickness maps. To date (PubMed Medline) this study involves the largest patient population examined, in which automatically measured choroidal thickness and volume are correlated with sex, age, refractive error, and axial length, not only in normal subjects but also in high myopia and hyperopia (from −22 diopter to +6 diopter).

Stepwise multiple regression analysis confirmed that choroidal thickness and volume, measured with a commercially available SS-OCT device, correlate with two independent variables, axial length, measured with optical low-coherence reflectometry, and age. The choroid both is the thinnest and has the smallest volume nasally. The focal increase of choroidal thickness at the fovea may be explained by increased metabolism.

EDI-OCT was earlier used to measure choroidal thickness. It has the highest sensitivity near to zero-delay and that sensitivity decreases for larger delays; an inversion of the OCT image was proposed, to move the zero-delay line closer to the choroid, providing enhanced sensitivity and increased imaging depth. Choroidal thickness can then be assessed with point-to-point manual caliper measurement taken on a single line scan, which is limited to the subfovea [9–11]. Some authors have suggested using the 6-line scanning protocol to obtain more information [12]. Volume measurement is obtained from compilation of a series of B-scans. To enable automated volume measurement the resolution of borders of the measured area must be clearly visible and distinguishable in all cases. Even if SD-OCT is able to provide retina volume measurements, no commercially available device is able to create choroidal thickness and volume maps. This is probably due to the fact that choroidoscleral boundary is not perfectly visible in all cases. As swept source OCT devices employ a longer light wavelength (1050 nm versus 840 nm in SD-OCT) they overcome much of the scattering of light on choroidal vasculature. SS-OCT obtains time-encoded information by sweeping a narrow-bandwidth laser through a broad optical spectrum. The backscattered intensity is detected with a photodetector and not with the spectrometers and CCD cameras used in SD-OCT devices. CCD cameras have a finite pixel size and thus there is a drop-off in signal with depth. Using photodetectors instead has led to a further increase in the potential resolution (1 *μ*m). The scan speed in swept-source instruments is twice that of SD-OCT devices (100,000 A-scans/sec compared to 50,000 A-scans/sec.). This enables faster acquisition of B-scans and a more accurate 3-dimensional image of the retina and choroid. It was earlier confirmed that despite the different wavelengths choroidal measurements performed with EDI-SOCT and SS-OCT are highly comparable [13].

This paper is the first to present automatic choroid thickness and volume measurements performed with a commercially available SS-OCT device in a wide range of patients in regard to age (15–79 years) and refractive error (−22 diopter to +6 diopter). The possibility of obtaining choroidal volume scans was presented before [14].

At 221 *μ*m the mean subfoveal choroidal thickness we measured with SS-OCT is lower than that previously reported in SD-OCT studies (272 *μ*m–354 *μ*m) and is lower than the results obtained with the prototype version of SS-OCT performed on Japanese subjects (354 *μ*m) [14].

However, the mean focal subfoveal choroidal thickness (choroidal thickness at the foveola) measured manually was 259 *μ*m, which is more comparable to the previous results mentioned above. The different results may be due to differences in how the measurements are taken. With the earlier SD-OCT machines and the SS-OCT prototype, choroidal thickness measurement is possible only manually at certain spots whereas we were additionally able to measure the mean subfoveal choroidal thickness in all 9 map sectors as defined by ETDRS. Thus, automatic foveal choroidal thickness measurement corresponds to an area with a diameter of 1000 *μ*m, centered on the foveola. The results we obtained may indicate that any increase in choroidal thickness is only focal and that thickness decreases with the distance from the foveola. Additionally in our group many myopic subjects were included. Another explanation may be that the difference is due to incorrect measurement by the automated software.

Our study confirms earlier SD-OCT and prototype SS-OCT reports that the choroid is thinnest on the nasal side of the fovea. Automatic measurement in certain sectors additionally enabled us to determine that this decrease reaches statistical significance about 1.5 mm from the foveola.

Moreover, this paper is the first to present quantitative measurement of choroidal volume. We succeeded in confirming that choroidal volume is lowest on the nasal side of the fovea, with statistical significance about 1.5 mm from the foveola. Choroidal volume in different ETDRS subfields is measured from different geometrical figures, thus central volume cannot be compared with volumes in the outer and inner rings. Choroidal volume in the fovea is the volume of a cylinder with an upper and lower diameter of 1000 *μ*m and the height of the cylinder is the foveal choroidal thickness (*V* = *πr* ^2^ *h*; *V*—cylinder volume, *r*—radius, and *h*—height). Choroidal volumes in the inner and outer quadrants are volumes of irregular geometrical figures with base diameters bigger than the foveal, which explains why the choroidal volume values in all subfields are bigger than in the center. Our SS-OCT study presents a mean subfoveal choroidal volume of 0.17 mm^3^, which is lower than in the earlier SD-OCT studies by Shin et al., who reported 0.24 mm^3^ [12].

Using multiple regression analysis, we demonstrated that choroidal thickness independently correlates with age and axial length. Correlation between choroidal thickness and age is well established. Autopsy studies have reported a 1.1 *μ*m decrease per year, previous SD-OCT studies have suggested 0.9 *μ*m–1.54 *μ*m per year, and early SS-OCT studies performed with a prototype device reported that the mean decrease is about 14 *μ*m every 10 years [13–17]. Our study presents a yearly mean decrease of 1.289 *μ*m. Our figure may be affected by the *R* ^2^ measurements in our study being as low as 0.08 which, in itself, confirms the great interindividual variability also reported by Ikuno et al. [15]. In our study for example, three 20-year-old patients had an axial length of 24 mm yet their central choroidal thickness varied from 288 *μ*m to 361 *μ*m. Ruiz-Moreno et al. on the other hand reported no differences in choroidal thickness between pediatric and older populations [18]. It may require further studies to determine which other factors are responsible for intraindividual changes in choroidal thickness. It may vary with race or other genetic predispositions or other unknown factors.

Regression analysis also revealed that choroidal thickness decreases 18.7 *μ*m with every decrease of 1 diopter (*R* ^2^ = 0.2). This is more than what Ikuno et al. proposed (9.3 *μ*m per diopter) perhaps because their analysis only included healthy subjects without high myopia whilst our group analyzed a wider spectrum of refractive errors (from −22 to +6 diopter).

Multivariate analysis by Ikuno et al. suggested that refractive error also independently correlates with choroidal thickness whereas we found no correlation. Again, this may be because Ikuno et al. included a low spectrum of axial lengths and refractive errors in their study and we investigated individuals from high myopia to hyperopia [15].

To conclude with, SS-OCT enables automatic creation of choroidal thickness and volume maps.

This study presents that choroid is at its thinnest nasally, about 1.5 mm from the fovea. Choroidal volume is also lowest on the nasal side.

Multivariate analysis confirmed that choroidal thickness independently decreases with increasing age and higher axial length.

## Figures and Tables

**Figure 1:** (a) Swept source OCT in a healthy volunteer. The red horizontal lines were drawn automatically at the inner and outer choroidal boundaries. The vertical line was drawn manually, to measure central choroidal thickness. (b) Swept source OCT fundus view. The circle and numbers are drawn automatically and represent automated thickness and volume measurements, which were performed in 9 segments according to early treatment diabetic retinopathy study.

**Figure 2:** Choroidal thickness (a) and volume (b) correlate negatively with age (*P* < 0.001).

**Figure 3:** Choroidal thickness (a) and volume (b) correlate negatively with axial length (*P* < 0.001).

**Table 1:** Choroidal thickness measurement.

	All (*μ*m) (mean age 43.2 years)	Emmetropia (mean age 44.7 years)	All myopic eyes (mean age 41.4 years)	High myopia (>6 Dptr) (mean age 42.6 years)	Hyperopia (mean age 56.9 years)
Fovea manually determined	259	326	231	187	312
Fovea automatically determined (1000 *μ*m diameter)	221	259	208	172	234.7
Inner ring (3 mm diameter)					
Superior	220	268	204	176	221
Inferior	214	252	200	159	233
Temporal	217	251	204	170	231
Nasal	202	240	188	157	221
Outer ring (6 mm diameter)					
Superior	231	280	211	176	265
Inferior	210	236	188	157	257
Temporal	216	247	204	174	228
Nasal	182	226	165	140	212

**Table 2:** Choroidal volume measurement.

	All (*μ*m^3^) (mean age 43.2 years)	Emmetropia (mean age 44.7 years)	All myopic eyes (mean age 41.4 years)	High myopia (>6 Dptr) (mean age 42.6 years)	Hyperopia (mean age 56.9 years)
Fovea automatically determined (1000 *μ*m^3^ diameter)	0.17	0.2	0.16	0.13	0.18
Inner ring (3 mm diameter)					
Superior	0.46	0.4	0.48	0.59	0.35
Inferior	0.34	0.4	0.31	0.25	0.37
Temporal	0.34	0.37	0.32	0.26	0.36
Nasal	0.31	0.4	0.29	0.24	0.35
Outer ring (6 mm diameter)					
Superior	1.2	1.47	1.12	0.94	1.4
Inferior	1.1	1.24	1.06	0.86	1.36
Temporal	1.1	1.3	1.0	0.91	1.2
Nasal	0.9	1.17	0.87	0.75	1.1

## References

[1] Spaide RF, Koizumi H, Pozonni MC (2008). Enhanced depth imaging spectral-domain optical coherence tomography. *The American Journal of Ophthalmology*.

[2] Manjunath V, Taha M, Fujimoto JG, Duker JS (2010). Choroidal thickness in normal eyes measured using cirrus HD optical coherence tomography. *The American Journal of Ophthalmology*.

[3] Barteselli G, Chhablani J, El-Emam S (2012). Choroidal volume variations with age, axial length, and sex in healthy subjects: a three-dimensional analysis. *Ophthalmology*.

[4] Michalewska Z, Michalewski J, Nawrocki J (2013). New OCT technologies take imaging deeper and wider. *Retinal Physycian*.

[5] Holzer MP, Mamusa M, Auffarth GU (2009). Accuracy of a new partial coherence interferometry analyser for biometric measurements. *The British Journal of Ophthalmology*.

[6] Chakraborty R, Read SA, Collins MJ (2011). Diurnal variations in axial length, choroidal thickness, intraocular pressure, and ocular biometrics. *Investigative Ophthalmology and Visual Science*.

[7] Michalewski J, Nawrocki J, Nawrocka Z, Dulczewska-Cichecka K, Nawrocki J Lamina suprachoroidea and suprachoroidal space delineating the outer margin of the choroid in swept-source OCT.

[8] Early Treatment Diabetic Retinopathy Study Research Group (1991). ETDRS report number 7: early treatment diabetic retinopathy study design and baseline patient characteristics. *Ophthalmology*.

[9] McCourt EA, Cadena BC, Barnett CJ, Ciardella AP, Mandava N, Kahook MY (2010). Measurement of subfoveal choroidal thickness using spectral domain optical coherence tomography. *Ophthalmic Surgery, Lasers & Imaging*.

[10] Imamura Y, Fujiwara T, Margolis R, Spaide RF (2009). Enhanced depth imaging optical coherence tomography of the choroid in central serous chorioretinopathy. *Retina*.

[11] Fujiwara T, Imamura Y, Margolis R, Slakter JS, Spaide RF (2009). Enhanced depth imaging optical coherence tomography of the choroid in highly myopic eyes. *The American Journal of Ophthalmology*.

[12] Shin JW, Shin YU, Lee BR (2012). Choroidal thickness and volume mapping by a six radial scan protocol on spectral-domain optical coherence tomography. *Ophthalmology*.

[13] Ikuno Y, Maruko I, Yasuno Y (2011). Reproducibility of retinal and choroidal thickness measurements in enhanced depth imaging and high-penetration optical coherence tomography. *Investigative Ophthalmology and Visual Science*.

[14] Hirata M, Tsujikawa A, Matsumoto A (2011). Macular choroidal thickness and volume in normal subjects measured by swept-source optical coherence tomography. *Investigative Ophthalmology and Visual Science*.

[15] Ikuno Y, Kawaguchi K, Nouchi T, Yasuno Y (2010). Choroidal thickness in healthy Japanese subjects. *Investigative Ophthalmology and Visual Science*.

[16] Ramrattan RS, van der Schaft TL, Mooy CM, de Bruijn WC, Mulder PG, de Jong PT (1994). Morphometric analysis of Bruch’s membrane, the choriocapillaris, and the choroid in aging. *Investigative Ophthalmology and Visual Science*.

[17] Margolis R, Spaide RF (2009). A pilot study of enhanced depth imaging optical coherence tomography of the choroid in normal eyes. *The American Journal of Ophthalmology*.

[18] Ruiz-Moreno JM, Flores-Moreno I, Lugo F, Ruiz-Medrano J, Montero JA, Akiba M (2013). Macular choroidal thickness in normal pediatric population measured by swept-source optical coherence tomography. *Investigative Ophthalmology and Visual Science*.

